# The Cataleptic, Asymmetric, Analgesic, and Brain Biochemical Effects of Parkinson's Disease Can Be Affected by *Toxoplasma gondii* Infection

**DOI:** 10.1155/2020/2546365

**Published:** 2020-05-01

**Authors:** Mahnaz Taherianfard, Moslem Riyahi, Mostafa Razavi, Zahedeh Bavandi, Narges Eskandari Roozbahani, Mohammad Mehdi Namavari

**Affiliations:** ^1^Physiology Division, Department of Basic Science, School of Veterinary Medicine, Shiraz University, Shiraz, Iran; ^2^Department of Pathobiology, School of Veterinary Medicine, Shiraz University, Shiraz, Iran; ^3^Pharmacology Division, Department of Basic Sciences, School of Veterinary Medicine, Shiraz University, Shiraz, Iran; ^4^Razi Vaccine and Serum Research Institute, Shiraz, Iran

## Abstract

**Purpose:**

Parkinson's disease (PD) is a neurodegenerative disorder with progressive motor defects. Therefore, the aim of the present investigation was to examine whether catalepsy, asymmetry, and nociceptive behaviors; the Nissl-body and neuron distribution; brain-derived neurotrophic factor (BDNF); malondialdehyde (MDA); total antioxidant capacity (TAC) levels; and the percentage of dopamine depletion of striatal neurons in the rat model of Parkinson's disease (PD) can be affected by *Toxoplasma gondii* (TG) infection.

**Methods:**

Fifty rats were divided into five groups: control (intact rats), sham (rats which received an intrastriatal injection of artificial cerebrospinal fluid (ACSF)), PD control (induction of PD without TG infection), TG control (rats infected by TG without PD induction), and PD infected (third week after PD induction, infection by TG was done). PD was induced by the unilateral intrastriatal microinjection of 6-hydroxydopamine (6-OHDA) and ELISA quantified dopamine, BDNF, MDA, and TAC in the striatum tissue. Cataleptic, asymmetrical, nociceptive, and histological alterations were determined by bar test, elevated body swing test, formalin test, and Nissl-body and neuron counting in the striatal neurons.

**Results:**

The results demonstrated that PD could significantly increase the number of biased swings, descent latency time, and nociceptive behavior and decrease the distribution of Nissl-stained neurons compared to the control and sham groups. TG infection significantly improved biased swing, descent latency time, nociceptive behavior, and the Nissl-body distribution in striatal neurons in comparison to the PD control group. The striatal level of BDNF in the PD-infected and TG control groups significantly increased relative to the PD control group. The striatal MDA was significantly higher in the PD control than other groups, while striatal TAC was significantly lower in the PD control than other groups.

**Conclusions:**

The current study indicates that TG infection could improve the cataleptic, asymmetric, nociceptive and behaviors; the level of striatal dopamine release; BDNF levels; TAC; and MDA in PD rats.

## 1. Introduction

Parkinson's disease (PD) is one of the most widespread neurodegenerative diseases, with a prevalence of approximately 1% of individuals with an age above 65 years [1]. It determined by the chronic and slowly progressive injury and depletion of dopaminergic neurons in the substantia nigra that may led to motor disturbances, including bradykinesia, akinesia, rest tremor, and postural instability. Likewise, patients may suffer from nonmotor symptoms, including depression, anxiety, rapid eye movement (REM) disorder, and pain [2, 3]. Catalepsy, the impairment of movement initiation, is an extrapyramidal dysfunction known as a prominent motor symptom of PD, which is related to the striatal dopamine reduction. Cataleptic behavior in the PD rodent has been employed as a standard model of bradykinesia and rigidity in human PD [4]. Pain is an important nonmotor symptom in PD patients that overshadow the quality of PD's life. Forty to 85 percentages of PD patients have painful sensations [3] in five different manners: musculoskeletal (related to parkinsonian rigidity and akinesia), neuropathic (related to neural lesion), dystonia-related, akathisia, and central neuropathic pain [5]. Although some genetic mutations identified have been associated with PD, the exact causes of PD remain unknown. Nevertheless, the crucial roles of oxidative stress and neuroinflammation in its pathogenesis have been well documented [6]. Even though the underlying cause of idiopathic PD remains unknown, the role of an increase in the oxidative stress, inflammatory responses, and mitochondrial dysfunction of dopamine neurons and a decrease in the availability of brain-derived neurotrophic factor (BDNF) have been well documented as pathophysiologic mechanisms [7].

*Toxoplasma gondii* (TG), a member of the phylum *Apicomplexa*, is an obligate intracellular parasite with high worldwide distribution which has infected one-third of the world population [8]. Tachyzoites, the invasive form of TG, infect neural cells. Afterward, in rodents, they differentiate into bradyzoites, which form the intracellular brain cysts. TG infection is considered asymptomatic in adults, but it can cause problems such as encephalitis, blindness, and mental retardation in immunocompromised individuals and congenitally infected children [8]. It has been observed that brain biochemistry is affected by the host immune system responses against TG infection [9]. On the other hand, TG protects itself and host cells against the immune response through some strategies, such as increasing the levels of antioxidant activity [10], brain-derived neurotrophic factor )BDNF( [11], dopamine concentration [12], and antiapoptotic activity [13]. IFN-*γ* production is increased by TG infection through tyrosine hydroxylase activity 1 (TH1) immune response [14]. Torres et al. found that TG reduces the expression of N-methyl-D-aspartate (NMDA) receptor via IFN-*γ* stimulation [15]. Moreover, TG activates the astrocytes that synthesize some metabolites to modulate NMDA receptor function [16]. The dopamine levels can be changed by TG in the brain [12]. The behavioral changes observed in infected rodents are attributed to its ability to change the neurotransmitter levels [12]. Dopamine depletion in PD decreases the inhibitory control of the corticostriatal glutamatergic pathway [17]. Moreover, PD causes hypofunction of the output pathways from the substantia nigra and medial globus pallidus, which leads to the increase in the excitatory subthalamic glutamatergic output [18].

Striatal medium spiny neurons contained dopamine D2 receptors, which are involved in controlling extrapyramidal functions. Haloperidol, an antipsychotic agent, induces catalepsy via selective blocking of dopamine D2 receptor in the striatum [19]. Previous findings indicated that the dopamine system has a modulatory effect on the pain and dopamine D2 receptor agonists attenuate nociceptive behavior initiation in animals and humans. Therefore, striatal dopamine enhancement can attenuate PD pain and catalepsy symptoms. There are a few investigations on the interaction of TG infection with PD pain symptom and behavioral changes; and these results are in paradox; also, most of the study on the relation between TG and PD were done according to a serological study in human and there is not any study on the brain. Therefore, the present investigation was done to study the effects of TG infection on experimental PD induction rat's asymmetric and cataleptic behavior, pain perception, percentage of dopamine depletion, level of striatal BDNF, TAC and MDA levels, and Nissl-body and neuron distribution in striatal neurons.

## 2. Materials and Methods

### 2.1. Subjects and Study Design

Fifty Sprague Dawley male rats, weighing 220–300 g in standard condition 12-h light/dark cycle with food and water ad libitum were used. Animal handling was conducted according to the Ethical Committee for Animal Experiments at Shiraz University. Animals were randomly divided into five groups (*n* = 10 in each group): control group, intact rats; sham group, intrastriatally ACSF-injected rats; PD control group, induction of PD in rats by intrastriatal injection of 6OHDA; TG control group, rats were infected by TG; and PD-infected group, the infection by TG was done on the third week after the induction of PD..

RH strain TG tachyzoites were obtained from the Razi Vaccine and Serum Research Institute, Shiraz, Iran. For infection induction, rats received intraperitoneal (IP) injection of 200 *μ*l normal saline containing 10^5^ tachyzoites (counted by a hemocytometer). At the end of the experiment, for the confirmation of tissue cyst formation, the brain smears were prepared and stained by Giemsa (Figure 1(a)).

### 2.2. Behavioral Testing

Rats were subjected to elevated body swing test by the method of Roghani et al. [20]. Catalepsy was evaluated by the bar test. In brief, the forepaws of each rat were located in a half-rearing position on a horizontal metal bar, which was set at 9 cm above the base in a parallel form. The time was recorded until the rats removed one paw from the bar (descent latency time). Descent latency cutoff time was 180 sec for the bar test [21]. The PD-infected design of the behavioral tests was performed in four steps: first, one week before the surgery; second and third, two and three weeks after surgery, respectively; and forth, eight weeks after TG infection (Figure 1(b)).

### 2.3. Formalin Test

Pain behavior was examined by the formalin test eight weeks after the infection as follows: the rats were located in the 32 × 32 × 32 cm Plexiglas boxes and a mirror was mounted at a 45^″^ angle, beneath the floor to the view of the rats' paws. 50 *μ*l of 2.5% formalin was injected by 27G needle into the foot plantar surface of the hind paw contralateral to the 6-OHDA injection site. The pain behavior was scored in 15 sec intervals and continued for 60 min [22]. After behavioral testing, the animals were decapitated and the striatum was dissected and stored at -80 C°.

### 2.4. Stereotaxic Surgery

Animal was anesthetized by IP injection of ketamine (100 mg/kg) and xylazine (8 mg/kg). PD induction was done by a unilateral and single injection of 20 *μ*g of 6-OHDA (in 4 *μ*l saline with 0.2 mg/ml of ascorbic acid) into the striatum (0.7 mm anterior to the bregma, 3 mm lateral to the midline, and 5 mm ventral to the dura).

The accuracy of the injection site location was determined by the microinjection of 4 *μ*l methylene blue into the striatum at the end of each experiment. In decapitated rats, the brains were removed and then were fixed in 10% of phosphate-buffered formalin for 24 hours. The striatum injection site was confirmed by comparing it with the atlas of Paxinos and Watson (Figure 1(c)).

### 2.5. Nissl Body and Neuron Distribution in the Striatum

At the end of the experiments, the rats were deeply anesthetized and sacrificed. For Nissl-body and neuron distribution measuring, after brain tissue fixation by 10% formalin, automatic tissue processor prepared paraffin blocks; then, 5 *μ* coronal section of the brain blocks in the region of striatum neurons was prepared. In all sections, Nissl-body counting in six cells and cell counting in six parts of each slide section of the striatum in all of the groups by Cresyl violet and hematoxylin eosin staining were done.

### 2.6. Dopamine, BDNF, TAC, and MDA Measurement

Dopamine concentration was measured using an ELISA kit (RE59161, IBL, Hamburg, Germany) in 50 *μ*g of homogenized striatal tissues based on Mabandla et al.'s modification [23]. The percentage of dopamine relative to the control group was determined according to following formula:

(1) $$\begin{array}{c} \frac{\text{dopamine concentration of group }x}{\text{dopamine concentration of control group}}\times 100 \end{array}$$

A rat ELISA kit (MyBioSource, USA, catalog # MBS824814) according to the manufacturer's instructions measured striatal BDNF. An ELISA standard kit was used to evaluate striatal TAC (ZB-TAC-96A, Zell Bio Germany) and MDA (ZB-MDA-96A, Zell Bio Germany).

### 2.7. Statistical Analysis

SPSS version 22 was used for data analysis. The Kolmogorov–Smirnov test was used for verifying the normalization of data. One-way ANOVA and Tukey's test, as the post hoc test, were used, and the significant level was considered *P* < 0.05.

## 3. Result

Catalepsy, via the bar test, revealed a significant increase in the descent latency time at the second, third, and fourth steps in the PD control group compared to the control and sham groups (*P* < 0.001). In addition, the PD-infected group showed a significant (*P* < 0.001) increase in the descent latency time at the second and third steps, but not at the fourth step. The TG control group had no significant difference in descent latency time in all steps in comparison with the control and sham groups (*P* > 0.05) (Figure 2(a)).

The elevated body swing test (EBST) confirmed asymmetric behavior representation and success of PD induction. It was performed at four steps of behavioral investigation as EBST1, EBST2, EBST3, and EBST4 (Figure 2(b)). As shown in Figure 2(b), the PD control and PD-infected groups showed a significant (*P* < 0.001) increase in the number of swinging in comparison to the control, sham, and TG control groups in EBST2 and EBST3. In EBST4, the PD-infected group revealed a significant reduction in the biased swing in comparison with the PD control group, whereas it had no significant difference with the control, sham, and TG control groups. However, the PD control group exhibited a significant increase in the biased swing compared with other groups.

As shown in Figure 3(a), after formalin injection into the hind paw, the PD control group showed a significant increase in the nociceptive scores in the early phase compared to the control and sham (*P* < 0.05) and TG control groups (*P* < 0.001). The PD-infected group had lower formalin-induced nociceptive scores in the early phase of the formalin test in comparison with the control and sham (*P* < 0.05) and PD control groups (*P* < 0.01). In the interphase of the formalin test, the PD control group showed a significant (*P* < 0.01) increase in the nociceptive scores in comparison to another groups, but there were no significant differences among the other groups (Figure 3(b)). As illustrated in Figure 3(c), the PD control group had a significant increase in the nociceptive scores in the late phase of formalin test compared to the other groups (*P* < 0.05).

As shown in Figure 4, a significant loss of Nissl-body in the striatal cells was evident in the PD control group compared with other groups (*P* < 0.001). Nevertheless, the PD-infected group significantly recovered from the Nissl-body loss in the striatal cells in comparison with the PD control group (*P* < 0.001). Meanwhile, no significant difference was found between the PD-infected and control, sham, and TG control groups (*P* > 0.05).

According to Figure 5 the number of neuron in striatum was significantly lower compared with other groups (*P* < 0.01). The PD-infected group significantly recovered from the neuron loss in the striatal cells in comparison with the PD control group (*P* < 0.001). Meanwhile, no significant difference was found between the PD-infected and control and sham groups (*P* > 0.05).

Table 1 shows that the percentage of dopamine in striatum neurons of the PD group is lower than that of the control; however, this reduction in the PD control was higher than that of the PD-infected group. Additionally, TG infection led to an increase in the mean of the dopamine concentration to 25.24% more than that of the control group.

BDNF of the striatum had a significant reduction (*P* < 0.001) in the PD control group compared to all the other groups (Figure 6(a)). The TG control group showed a significantly higher level of BDNF compared to the PD infected (*P* < 0.01), but PD infected had no significant differences with the control and sham groups (*P* > 0.05).

Figure 6(b) showed that the PD control group significantly decrease the TAC levels compared to the control and sham groups (*P* < 0.05), whereas the PD-infected and TG control groups showed no significant decrease in TAC levels vs. the control and sham groups (*P* > 0.05).

Figure 6(c) showed that the PD control group significantly increased the MDA levels compared to the control and sham groups (*P* < 0.001) whereas the PD-infected and TG control groups showed no significant increases in MDA levels vs. the control and sham groups (*P* > 0.05).

## 4. Discussion

The aim of the present study was to investigate the effect of the cataleptic and analgesic behaviors of the rat model of PD and how they may be affected by TG infection. Catalepsy is an extrapyramidal dysfunction that is explained as a disability to improve the external abnormal forced positions [24]. In addition to motor symptoms, pain is one of the most troublesome nonmotor symptoms of PD with a high prevalence that impairs patients' quality of life.

In our experiment, no significant asymmetry and descent latency time were observed among groups in the first step of the behavioral test. Following progressive dopaminergic nigrostriatal degeneration and decrease in the ipsilateral dopamine level, this imbalance resulted in a functional asymmetry [25]. In agreement with the previous studies, the results of this study indicated that PD induction significantly increase the biased swings in the second and third steps of the behavioral test compared with the other groups [20, 25–27]. In the PD-infected group, a significant decrease in the biased swing was observed in the fourth step of the behavioral test compared to the PD control group. TG was able to encode an enzyme with TH activity, a tyrosine to L-DOPA converter, which, in turn, is the rate-limiting step of the dopamine synthesis [28]. As shown in the results, the PD control group caused dopamine depletion by 84.53% in the striatum tissue. The degree of striatum DA reduction in PD-infected rats was 36.27%; as a result, TG infection has prevented severe dopamine decrease in the striatum. Additionally, the TG control group showed 25.24% of dopamine amplification in the striatum. In agreement with our finding, an increase for dopamine in the different regions of infected mouse brains including the striatum has been reported [11]. Decreasing dopamine in the lesioned striatum has been known as the primary factor of cataleptic behavior with concomitant descent latency [29]. Induction of PD causes damage to the nigrostriatal dopaminergic neurons, resulting in the abnormal firing of the basal ganglia circuits, manifested as muscle rigidity and catalepsy. Our results were consistent with those of other studies and showed that the descent latency time increased in the 6-OHDA-lesioned rats compared with other groups [30, 31]. However, PD-infected rats showed a significant decrease in descent latency.

Similar to the previous studies, in our experiment, in the PD control group, dopamine depletion increased formalin-induced pain behaviors in all three phases of the formalin test compared with the other groups [3, 5]. Hence, it can be concluded that the nigrostriatal dopaminergic system plays an important role in the processing of pain behavior. Previous studies have shown that the intrastriatal injection of dopamine D2 receptor agonists inhibits pain responses [32]. Present results were in agreement with a report that brain dopamine levels increased by TG infection [33]. TG infection improved PD-induced hyperalgesia and rats exhibited less pain behavior compared to the control, sham, and PD control groups in the early phase, interphase, and late phase of the formalin test.

Diminution of the asymmetric behavior following TG infection probably indicates its potency in increasing the striatal dopamine at a level that attenuates motor bias. It has been shown that the increase in the dopaminergic neuron activity and dopamine release could attenuate the catalepsy induced by PD [30]. Striatal medium spiny neurons, in addition to dopaminergic projections from the substantia nigra (inhibitory pathway), receive the glutamatergic input (excitatory pathway) from the motor cortex [34]. Previous research have indicated that the decrease in the function of glutamatergic neurons or NMDA-selective glutamate receptor within the striatum could lead to a reduction in the catalepsy of PD patients [35]. Hama et al. found that NMDA agonist receptors involved in the maintenance of hyperalgesia and NMDA antagonists have analgesic effects on the management of hyperalgesia [36]. Kynurenic acid is an endogenous NMDA-receptor antagonist with antiexcitotoxicity activity in the brain. Schwarcz and Hunter showed that TG infection could increase the synthesis of kynurenic acid in the brain via an immune process [16]. The effectiveness of kynurenic acid in the relief of pain has been confirmed in recent studies [37]. It could be a possible explanation for our observations, where in the fourth step of behavioral test, the PD-infected rats revealed a significant attenuated cataleptic and pain behavior. In the present study, it seems that TG via increasing striatal dopamine and decreasing glutamate through NMDA receptor exerts anticataleptic and analgesic effects on PD rats.

Meanwhile, in present study, the Nissl-body and neuron distribution in the ipsilateral striatum to the site of 6-OHDA injection have shown significant reduction in the Nissl-body of striatum neurons in the PD control group compared to the other groups; whereas, no significant differences were observed between the PD-infected, control, and sham groups. Therefore, TG could compensate for the decrease in the Nissl-body and neuron numbers induced by PD in the rats' striatum neurons.

Brain-derived neurotrophic factor (BDNF) is a member of the nerve growth factor (NGF) with a critical role in neuronal development, survival, and plasticity that is reduced in PD's brain [38]. Previous studies have demonstrated that BDNF could play a primary role in the protection of dopaminergic neurons against neurotoxins [39]. Present results revealed that TG infection could increase striatal BDNF level in PD-infected rats in comparison with the PD control rats. Therefore, TG recovered neurons against the neurotoxicity of 6-OHDA, probably due to improving striatal BDNF level. Consistent with our results, Xiao et al. reported that TG could increase the BDNF levels in infected mouse striatum tissue. They also demonstrated microRNA- (miR-) 132 high expression in the striatum of infected mice [11]. Transcription of miR-132 in neuronal cells is upregulated by BDNF; it seems that miR-132 mediated the effects of BDNF on the brain [40]. Therefore, miR-132 plays important roles in neurogenesis, synaptic plasticity and neuronal differentiation, neuronal outgrowth, and sprouting [41]. It regulates the differentiation of dopamine neurons from mouse embryonic stem cells [42]. Consequently, it seems that BDNF protects dopaminergic neurons against oxidative stress and prevents cell death [39]. It seems that TG protects cells against oxidative stress via increasing the BDNF levels.

Present findings showed a significant increase in the levels of striatal MDA and decrease in the TAC levels in the PD control group rats compared with the control and sham groups. TG is able to express an antioxidant system, including superoxide dismutase, catalase, at least one peroxiredoxin and complete thioredoxin, and glutathione-based antioxidant systems, that could protect cells against reactive oxygen species (ROS) [43]. An in vitro study by Zhou et al. showed that *TG* infection caused a significant reduction of NADPH oxidase 4 (Nox4) mRNA and protein level and intracellular reactive oxygen species (ROS) level of the host. These results suggest that Nox4 is the main target for *TG* in reducing host intracellular ROS level, and PI3K/Akt signaling pathway is responsible for the suppression of Nox4 expression. The results are consistent with our in vivo results in oxidative stress [44].

## 5. Conclusion

Present investigation revealed that TG infection might repair cataleptic, asymmetric, and pain behaviors in the PD control rats by the following ways: (1) enhancing the release of dopamine in the striatum, (2) inhibiting the NMDA-selective glutamate receptor within the striatum by increasing the synthesis of kynurenic acid and improving the striatal BDNF level of the rescued neurons against 6-OHDA, and (3) enhancing the TAC levels and decreasing the MDA levels. Further studies are required for a deeper understanding of the proposed pathways responsible for the anticataleptic, antiasymmetric, antinociceptive, and biochemical changes, which are associated with the TG infection in the PD rats. The results of the present study can be used for the development of new drugs or vaccine for the treatment of Parkinson's disease.

## Figures and Tables

**Figure 1:** (a) Photomicrograph showing *Toxoplasma gondii* cysts (Giemsa stained) in a brain smear of infected rats. (b) The overall design of the study and the scheduling of behavioral tests. (c) Photomicrograph shows the rat brain section in the striatum region confirming the injection site.

**Figure 2:** Two behavioral tests for PD induction confirmation. (a) Bar test (sec) and (b) EBST test in all groups. ^∗^*P* < 0.05, ^∗∗^*P* < 0.01, and ^∗∗∗^*P* < 0.001 significant differences. Data are shown as means ± SEM.

**Figure 3:** Nociceptive score in the PD-infected rats. (a) The mean of nociceptive score in the early phase of the formalin test. (b) The mean of the nociceptive score in the interphase of the formalin test. (c) The mean of the nociceptive score in the late phase of the formalin test. ^∗^*P* < 0.05, ^∗∗^*P* < 0.01, and ^∗∗∗^*P* < 0.001 significant differences. Data are shown as means ± SEM.

**Figure 4:** The total number of Nissl-bodies in rat striatum cells. ^∗∗∗^*P* < 0.001 significant difference. Data are shown as means ± SEM.

**Figure 5:** The number of neurons in the striatum (a). Photomicrograph of striatum neuron staining by hematoxylin eosin in the control group (b), sham group (c), PD control group (d), TG control group (e), and PD-infected group (f). ^∗∗^*P* < 0.01; ^∗∗∗^*P* < 0.001 significant differences. Data are shown as means ± SEM.

**Figure 6:** (a) Brain-derived neurotrophic factor (BDNF) protein concentration of striatum tissue. (b) Total antioxidant capacity (TAC) of striatum tissue. (c) Malondialdehyde (MDA) levels of striatum tissue. ^∗^*P* < 0.05, ^∗∗^*P* < 0.01, and ^∗∗∗^*P* < 0.001 significant differences. Data are shown as means ± SEM.

**Table 1:** Percentage of dopamine reduction relative to the control group.

Groups	Percentage of dopamine relative to control group
Control	100%
Sham	97%
PD control	15.45%
TG control	+125.24%
PD infected	63.73%

## Data Availability

The data used to support the findings of this study are available from the corresponding author upon request.
